The article "Study on Medication Rules of Traditional Chinese Medicine in Treating Constipation through Data Mining and Network Pharmacology" was published in 2022. Journal: Biomed Res Int.

# Study on Medication Rules of Traditional Chinese Medicine in Treating Constipation through Data Mining and Network Pharmacology

**DOI:** 10.1155/2022/6733851

**Published:** 2022-10-11

**Authors:** Shu-Min Xu, Li-Peng Bai, Jin-Gen Lu, Qing-Jun Dong, Bo Cao

**Affiliations:** ^1^Shanghai University of Traditional Chinese Medicine, Shanghai 200000, China; ^2^Department of Anorectal Traditional Chinese Medicine, the First Medical Centre, General Hospital of Chinese PLA, Beijing 100036, China; ^3^Department of Coloproctology, Longhua Hospital Shanghai University of Traditional Chinese Medicine, NO.725, South Wanping Road, Xuhui District, Shanghai 200032, China; ^4^The First Affiliated Hospital of Guizhou University of Traditional Chinese Medicine, Guiyang 550000, China

## Abstract

**Background:**

To explore the rules of TCM medication in the treatment of constipation in network pharmacology.

**Methods:**

Collect and screen the clinical intervention literature on TCM for constipation from China's national knowledge infrastructure, Wanfang and VIP databases established a database of TCM for constipation, applied R software (3.3.1) to analyze the pattern of prescriptions for TCM for constipation, and summarized the core prescription. The effective active compounds and action targets in the core prescription were screened by Traditional Chinese Medicine Systems Pharmacology (TCMSP) and Traditional Chinese Medicine Integrated Databases (TCMID), constipation-related targets were derived from the DisGeNET and GeneCards databases, Protein-protein interaction network (PPI) was drawn by STRING database, and enrichment analysis was conducted by the Clusterprofiler package in R software (3.3.1). Finally, molecular docking was used to validate the binding ability of candidate compounds to potential targets.

**Results:**

Two hundred sixteen target prescriptions were screened through data mining, involving 226 herbs. Association rule analysis results suggested that the “Angelicae sinensis-Radix-dried rehmanniae-Cistanche deserticola-Atractylodes macrocephala-Astragali Radix” was a strong affinity for medicine. Network pharmacology analysis of the core prescription resulted in the screening of 115 candidate compounds, such as quercetin, kaempferol, mangostin, eugenol A, and beta-sitosterol; 131 potential targets, such as PTGS2, PTGS1, and CHRM3; and 160 signaling pathways, such as lipid and atherosclerosis, proteoglycans in cancer, hepatitis B, Kaposi's sarcoma-associated herpesvirus infection, and PI3K/AKT pathways. Molecular docking showed that PTGS1-formononetin, PTGS2-kaempferol, and CHRM3-kaempferol were all well bound and well matched.

**Conclusions:**

This study provides a new method and ideas for clinical applications of integrated Chinese and western medicine in treating constipation.

The article "Study on Medication Rules of Traditional Chinese Medicine in Treating Constipation through Data Mining and Network Pharmacology" was published in 2022. Journal: Biomed Res Int.

## 1. Background

Constipation is one of the most common digestive system diseases in China. It mainly is manifested as the reduced number of defecation, laborious defecation, dry stool knot, and frequent cathartic use. Recently, the incidence of constipation in China has increased, and the long-term frequently serious defecation disorder reduced the quality of life. Currently, the main clinical treatment of constipation is the laxative and stimulant drug [1], but the long-term use of laxative drug will cause adverse effects, such as black colon, dry mouth, drug dependence, and gastrointestinal discomfort, and even increase the risk of intestinal obstruction and colon cancer [2–4].

TCM treatment emphasizes a holistic approach, taking into account both the symptoms and the root causes, and follows a discernment-based approach to treatment, overcoming the shortcomings of palliative treatment in Western medicine, which has unique advantages in improving the body's internal environment, reducing toxicity, and increasing effectiveness [5]. In addition, current traditional Chinese medicine- (TCM-) related research mainly focuses on experience summarization. These lack the in-depth study of the rules and mechanisms of medication in prescriptions. We urgently need to summarize the rules for the administration of Chinese medicine and analyze the mechanism of action of the herbs to provide the basis for the optimization of drug use and the screening of new compounds. Therefore, mining relevant information and medication laws from a large number of TCM data can not only be used to promote clinical drug use norms but also solve practical problems, such as new drug research and development, which can help to realize the inheritance and development of TCM treatment of constipation [6].

In this study, data mining was used to analyze the application rules of TCM in the treatment of constipation. We also proposed a computational systems pharmacology method and molecular docking to determine the associated molecular mechanisms. We intended to explore TCM's drug use pattern for treating constipation by collating the published clinical intervention literature of TCM in treating constipation, analyzing the frequency of drug use, nature, and taste of prescriptions. Using R software (3.3.1) to explore the key points of treatment and prescription use and the core combination of drugs [7], and using network pharmacology and molecular docking to explore potential active ingredients, core targets and main signaling pathways, elucidating the mechanism of action of traditional Chinese medicine in the treatment of constipation, providing reference value for further animal experiments and providing new ideas for the future clinical treatment of constipation. This, in turn, confirms the generalisability of the core prescription. The flow chart of this study is shown in Figure 1.

The article "Study on Medication Rules of Traditional Chinese Medicine in Treating Constipation through Data Mining and Network Pharmacology" was published in 2022. Journal: Biomed Res Int.

## 2. Materials and Methods

### 2.1. Prescription Mining

#### 2.1.1. Data Source

We conducted an electronic search of the Chinese databases from their inception to 31/12/2021. We searched the Chinese literature in CNKI, Wanfang, and VIP databases. All clinical intervention literature on the internal treatment of constipation with TCM was considered. The following search terms were used in combination: “Chinese medicine,” “traditional medicine,” “herbal medicine,” “herb,” “plant,” “prescription,” “decoction,” and “constipation,” among others.

#### 2.1.2. Study Selection

The inclusion criteria were as follows:

1. The included literature for this study had to be a clinical intervention case
2. The included literature was related to the internal use of TCM for constipation
3. The composition and dosage of the prescribed medication in the literature must be fully documented
4. The literature on the experience of famous veteran Chinese medicine practitioners can also be included in this study

The exclusion criteria were as follows:

1. Studies with cellular, animal, and other basic studies, reviews, meta-analysis, systematic evaluations, literature data mining, and mechanistic theoretical discussions
2. Duplicate publication, only abstract or lack of outcome data, and no access to obtain the full text
3. Constipation due to or in combination with other types of disease, e.g., tumour, pregnancy, radiotherapy, fractures, drug-related, and constipated irritable bowel syndrome
4. The combination of Western medicine taken orally or topically with acupuncture or enemas for constipation is in the literature

#### 2.1.3. Data Extraction and Collation

Following the search, all identified citations were collated and uploaded into EndNote (X9) citation manager, and duplicates were removed. The titles and abstracts were then screened against the inclusion criteria. Those studies meeting the eligibility criteria were retrieved in full. The full texts of selected studies were assessed in detail, and those that did not meet the inclusion criteria were excluded.

Relevant data were extracted from the final inclusion literature that included the review using a standardized data extraction template developed using a Microsoft Excel workbook. Double data extraction and entry were performed to ensure accuracy.

The names of herbs were standardized concerning the 2015 Chinese Pharmacopoeia (CHP) [8] and the 2016 Chinese Materia Medica (CMM) [9], the frequency of herbs and their ascription and taste were counted, and two people checked the results to establish a database. Any disagreements were resolved through discussion with the two primary reviewers and a third reviewer.

The article "Study on Medication Rules of Traditional Chinese Medicine in Treating Constipation through Data Mining and Network Pharmacology" was published in 2022. Journal: Biomed Res Int.

#### 2.1.4. Statistical Analysis

This study used R software (3.3.1) to perform a statistical analysis of the literature included in the database.

1. The normalized TCM was quantified by dichotomizing them using the Reshape function to build a shaping database
2. The ggplot2 function was applied to the data for frequency analysis to create a bar chart of Chinese medicines plotted
3. The Corrplot function was used to correlate the data and extract the core prescription. Association analysis was performed using rules and rules viz functions to visually demonstrate the degree of association used in TCM
4. This study uses *K*-means, PAM, and GMM algorithms to cluster the data

### 2.2. Network Pharmacology

The chemical components and related targets of the core prescription should be retrieved from the TCM Systems Pharmacology (TCMSP) Database (http://tcmspw.com/tcmsp.php) and TCM Integrative Database (TCMID) (http://www. http://megabionet.org/tcmid/) [10, 11]. The rules are as follows: oral bioavailability (OB) was set at 20%, and drug-likeness (DL), was set at 0.1 as the limiting screening condition for obtaining the core prescription active ingredient according to the pharmacokinetic rules [12, 13]. The UniProt database (https://www.uniprot.org/) is used to query the gene name of the target protein [14].

Using “constipation” as the keyword, the DisGeNET and GeneCards databases searched and screened the disease target genes [15–17]. The Venny map (Venny 2.1) is drawn to get the intersection target of the core prescription and constipation, which can be used as the potential target of the core prescription in treating constipation.

#### 2.2.1. Build an “Active Component-Action Target Network Map”

The active components of the core prescription and the related targets and the target genes of constipation were input into the Cytoscape 3.7.2 software to build a network map of the active component-action target network and clarify the potential interaction between the constipation target genes and the active components of the core prescription [18].

#### 2.2.2. PPI (Protein-Protein Network) Construction

Chemical components and intersection targets of the core prescription were imported into Cytoscape 3.7.2 software to construct the active component target network, and the topological properties of the network were analyzed; the intersection targets were uploaded to STRING database, and the species was limited to “human”; the confidence was 0.4, the free nodes were deleted, and the PPI network was constructed.

The article "Study on Medication Rules of Traditional Chinese Medicine in Treating Constipation through Data Mining and Network Pharmacology" was published in 2022. Journal: Biomed Res Int.

#### 2.2.3. GO and KEGG Pathway Enrichment Analysis

Furthermore, the Clusterprofiler package in R software (3.3.1) was used for the Gene Ontology (GO) enrichment analysis and Kyoto Encyclopedia of Genes and Genomes (KEGG) enrichment analysis of the core prescription acting targets, and the bioinformatics platform was used for visualization analysis of biological functions and pathways. *P* value ≤ 0.05 was used to screen biological functions and signal pathways of the core prescription acting targets.

### 2.3. Molecular Docking

To assess the credibility of the connection between the target and the compound and identify the core prescription for constipation treatment, molecular docking of the core compounds with core targets was carried out. Molecular docking can study the active components of the core prescription and its related targets in the treatment and can explain the mechanism of action and binding activity of active components and target proteins to a certain extent. Then, we run Schrodinger software for molecular docking and use PyMOL 2.1 to analyze the docking conformation visually.

## 3. Results

### 3.1. Prescription Statistics and Analysis

#### 3.1.1. Inclusion in the Literature

A total of 11,386 pieces of literature were initially searched including 2,978 on the CNKI database, 5,552 on Wanfang the database, and 2,856 on the VIP database. The following steps are as follows: (1) the literature was first checked against title and author to remove duplicates. (2) After that, the title and abstract were read for initial screening to eliminate irrelevant literature. (3) The full text of the literature was further read and rescreened to eliminate those not meeting the inclusion criteria. (4) Next, the literature was extracted from the prescriptions, and those with duplicate use of drugs and no clear prescription information were excluded.

#### 3.1.2. Analysis of the Frequency and Efficacy of TCM

Bar graph of 31 TCM used >30 times and classified according to the 2016 edition of traditional Chinese medicine. Bar graph of 31 TCM used >30 times is classified according to the 2016 edition of Traditional Chinese Medicine. The results showed that TCM for constipation is mainly tonic for deficiency, followed by qi regulating and diarrhea medicines, and the top 10 TCM in high-frequency combinations are mostly sweet tasting and warm in nature; they belong to the spleen and lung meridian. The overall treatment reflects the principle of tonifying deficiency, guiding stagnation, and clearing the bowels, which is in line with the basic pathogenesis of constipation in TCM theory. The medicine characteristics and TCM theory “deficiency of the internal organs” are shown in Figure 2.

The article "Study on Medication Rules of Traditional Chinese Medicine in Treating Constipation through Data Mining and Network Pharmacology" was published in 2022. Journal: Biomed Res Int.

#### 3.1.3. “Drug-Drug” Correlation Analysis

The Pearson correlation coefficient in the R software was used to measure the correlation between two random variables, i.e., the magnitude of the coefficient is directly proportional to the degree of correlation between the pairs. The larger the correlation coefficient is, the stronger the correlation between the two drugs. The top 64 herbal pairs with high correlation coefficients were extracted, e.g., *Atractylodis macrocephalae*-Bai Shao, rhubarb-*Angelicae sinensis*, *Herba cistanches*-firenuts, Radix *Rhizoma gastrodiae*-Mai Dong, and Radix *Astragali*-licorice (see Figure 3).

#### 3.1.4. “Drug-Drug” Association Analysis

The strength of association analysis is measured by support, confidence, and lift. The analysis of strong association rules for treating constipation using TCM in R software was set with minimum support of 0.1 and minimum confidence of 0.8. A total of 172 association rules were obtained, all with a lift of >1, which were considered valid. Among them, there were 12 association rules for two drugs, 75 association rules for three drugs, and 85 association rules for four drugs. The rules were ranked according to the support degree, and the top 10 drug pairs were extracted (see Tables 1–3).

The Apriori algorithm was applied for association rule analysis [19, 20], and the association rule graph was generated by selecting the highest support and confidence level. The confidence in the graph is the size of the circle, the elevation is the color shade, and the arrows represent the pointing relationship. From this graph, the darker the color and width of the line segments between two medicines, the thicker the relationship between these two medicines, and the lighter the line segments, the weaker the rules. Combined with the support and confidence analysis, TCM with more obvious lines in the graph are *Angelica sinensis*, Radix Rhizoma ginseng, *Herba cistanches*, Rhizoma *Atractylodis macrocephalae*, and Radix *Astragali*, and this graph is consistent with the results of the association rule (see Figure 4).

#### 3.1.5. Cluster Analysis

The *K*-means, PAM, and GMM algorithms of the R software clustering algorithm were used to cluster the drugs in the databases, which were set to cluster into 3 classes, and the results were presented through the dendrogram hierarchy. Based on the *K*-means algorithm, the optimal number of clusters was tested for 64 medicines with frequencies >5 times, and the results suggested that the best clustering results were obtained when the number of clusters was 2 (see Figure 5(a)).

The article "Study on Medication Rules of Traditional Chinese Medicine in Treating Constipation through Data Mining and Network Pharmacology" was published in 2022. Journal: Biomed Res Int.

Based on the PAM algorithm, the optimal number of clusters was tested on 64 medicines with frequencies >5 times, and the results suggested that the best clustering results were obtained when the number of clusters was 2 (see Figure 5(b)). By performing hierarchical clustering and drawing a tree diagram on the basis of the above association rule results for 64 medicines used >5 times, this study classified the results of the clustering analysis into two categories with similar drug characteristics according to the PAM algorithm, and the results suggested 48 Chinese medicines in category 1 and 16 medicines in category 2 (see Figure 5(c)).

Based on the GMM algorithm, the optimal number of clusters was tested on 64 medicines, and the best results were obtained when the number of clusters was 3 or 4 (see Figure 5(d)). According to the GMM algorithm, the tree diagram was divided into 3 categories with similar drug characteristics, and the results suggested 48 medicines in category 1, 10 medicines in category 2, and 6 medicines in category 3 (see Figure 5(e)). According to the GMM algorithm, the tree diagram was divided into 4 categories with similar drug characteristics, and the results suggested that there were 48 medicines in category 1, 10 medicines in category 2, 3 medicines in category 3, and 3 medicines in category 4 (see Figure 5(f)).

### 3.2. Network Pharmacology

#### 3.2.1. Screening of Active Components and Targets in Constipation

Using TCMSP and TCMID databases, 115 active components and 507 active targets were selected to establish the target protein database of drugs. Then, using the DisGeNET and GeneCards databases, a total of 1118 target genes related to constipation were retrieved using the keyword “constipation”. All targets of the drug were deduplicated and integrated to obtain potential targets of drug action for the treatment of constipation by mapping drug targets to disease targets using the Venny 2.1 (see Figure 6(a)).

#### 3.2.2. Construction of the PPI Network

The STRING database was used to construct the PPI network of target protein interactions for potential targets of drug pairs for the treatment of constipation and to obtain the structural and functional interactions between the proteins of interest and the genes.

The key genes in the PPI network were then obtained by Cytoscape 3.7.2 software. There are 131 key targets and 4656 connecting lines in the graph. The redder the color, the larger the node, and the greater the target degree value; i.e., these targets may have a strong correlation with constipation (see Figure 6(b)).

The article "Study on Medication Rules of Traditional Chinese Medicine in Treating Constipation through Data Mining and Network Pharmacology" was published in 2022. Journal: Biomed Res Int.

#### 3.2.3. GO Function Enrichment Analysis and KEGG Pathway Enrichment Analysis

In order to clarify the characteristics of the relevant targets of the key active components of the core prescription, GO and KEGG pathway enrichment analyses were performed in Figure 6(c). DAVID 6.8 (https://david.ncifcrf.gov/) is an online biological information repository and analysis tool for extracting biological information regarding gene functional annotation and pathways enrichment. These targets existed in the nucleus, cytoplasm, and plasma membrane of cells and were involved in biological processes, such as transcriptional regulation, drug response, signal transduction, cell proliferation, and senescence. The molecular function of these genes was involved in binding proteins, enzymes, and zinc ions. In GO enrichment analysis, 2352 GO items, 2133 biological processes, 80 cellular components, and 139 molecular function-related items were identified. KEGG enrichment analysis indicated that 160 pathways were affected by the active components of the core prescription with the smallest *P* value. The top 20 pathways included lipids and atherosclerosis, proteoglycans in cancer, hepatitis B, Kaposi's sarcoma herpesvirus infection, and PI3K-AKTB pathways. Based on this information, the core prescription compound-target-pathway network association was established.

#### 3.2.4. Construction of the Active Ingredient Target Network

The active component target network of constipation consists of 199 compound nodes, 131 target nodes, and 1202 edges. As shown in Figure 6(d), the core prescription has multicomponent and multitarget characteristics in treating constipation. The same active component can act on different targets, and the same target can also correspond to different active components.

### 3.3. Molecular Docking

#### 3.3.1. Molecular Docking Verification of Core Components in Constipation

The molecular docking results obtained according to the SP method are shown in Table 4. Additional complexes of proteins with small molecules were visualized by PyMOL 2.1 as described in Figure 7.

#### 3.3.2. Analysis of the Interaction between the Compound and the Protein

To better understand the interactions between the compounds and target genes, we constructed an interaction network between the key target genes and corresponding active compounds in the core prescription (Table 4). According to the compound-putative analysis results, the key compounds were quercetin, kaempferol, formononetin, diincarvilone A, and beta-sitosterol. To further explore the interactions between key compounds and key target genes, we performed molecular docking by PyMOL 2.1 software. We used PTGS1, PTGS2, and CHRM3 proteins to dock with quercetin, kaempferol, formononetin, diincarvilone A, and beta-sitosterol, as shown in Figure 7. Therefore, the binding pattern of formononetin to the PTGS1 protein is well displayed, so the compound is a potentially active small molecule. Several other compounds (quercetin and kaempferol) exhibited excellent binding patterns and docking scores with PTGS1, PTGS2, and CHRM3 target proteins and were well matched to the active site pockets of the proteins to form stable complexes with them.

The article "Study on Medication Rules of Traditional Chinese Medicine in Treating Constipation through Data Mining and Network Pharmacology" was published in 2022. Journal: Biomed Res Int.

## 4. Discussion

In recent years, people have paid more and more attention to the modernization, inheritance, and development of TCM. With the arrival of the era of big data and the rise of artificial intelligence, many software and platforms have emerged for TCM prescription analysis. Many medical researchers have devoted themselves to mining literature and data, hoping to guide clinical guidance better and give full play to the advantages of TCM. This study used data mining and R software [15, 16] to find the drug compatibility rules for constipation, determine the final core prescription, combine the network pharmacology and molecular docking [17, 23, 24], initially discuss the active ingredients and mechanism of core prescription for constipation, and provide new ideas for clinical and basic research.

In this study, in data mining in R software combined with the numerical ranking of support, confidence, and improvement, we can see that the core prescription of “Angelicae sinensis-Radix-dried rehmanniae-Cistanche deserticola-Atractylodes macrocephala-Astragali Radix” has high frequency and high comprehensive score and has good correlation. TCM treats constipation to fill and through. Angelica can nourish the blood and dryness; baishu can improve the qi and spleen; astragalus can benefit qi and aphrodisiac; angelica and astragalus can replenish qi, blood, and laxative; astragalus and baishu can play a role in rationalizing qi and laxative; cistanche can supplement kidney yang, improve muscles and activate blood, and run laxatives; raw yellow can nourish yin and moist intestines. The combination and use of the above drugs reflect the treatment of constipation to supplement qi and blood, regulating qi and guiding stagnation, nourishing Yin, and moistening dryness, which is in line with the basic pathogenesis of the “virtual standard” of constipation. As a basic Chinese medicine, the core prescription is widely found in multiple prescriptions to treat constipation, such as Runchang pills, Huangqi decoction, and Xinjia Huanglong decoction, which proves that the core prescription conforms to the clinical reality and is commonly used to treat constipation, and the data mining results are reliable.

The article "Study on Medication Rules of Traditional Chinese Medicine in Treating Constipation through Data Mining and Network Pharmacology" was published in 2022. Journal: Biomed Res Int.

Based on data mining and collation results, this study applied network pharmacology to investigate the mechanism of action of the core prescription for treating constipation and constructed a network between the effective compounds of the core prescription and the constipation-related genes. The network map analysis determined a total of 115 active components and 131 targets involved in the network construction. The compound-target network map can be predicted that the treatment-related components are quercetin, kaempferol, hilanin, and other activities. Quercetin is a flavonol compound with multiple bioactivities and widely found in natural plants and has antioxidation and anti-inflammatory effects. Quercetin relieves the symptoms of difficult defecation, reduces the harmful flora, and reduces the intestinal mucosa [25]. Kaempferol, a natural polyphenolic compound abundant in fruits, vegetables, and Chinese herbal medicine, has been used as one of the key research compounds for cancer, diabetes, and cardiovascular and cerebrovascular diseases. Naempferol improves the antioxidant capacity of the intestine and improves the laxative function in rats [26]. Manganin, a compound similar to estrogen, is extensively metabolized in rat intestinal flora. Studies have found that an effect on the balance of intestinal bacteria and imbalance of intestinal flora is one of the main causes of constipation [27, 28]. The above compounds have been shown to be an important component in constipation studies [29].

From the “core prescription-active, ingredient-target of action map” and the PPI network of key targets of the core prescription for constipation, the abnormal targets of the core prescription for constipation can be predicted, among which the closest relationships are with cyclooxygenase 2 (PTGS2), cyclooxygenase 1 (PTGS1), and acetylcholine receptor M3 (CHRM3). PTGS is a cyclooxygenase (COX); it has two isozymes [30, 31]: one is a structural type (PTGS1, COX-1), and the other is an inducible type (PTGS2, COX-2 ), which have similar basic protein structures and are all closely related to intestinal tumorigenesis [29]. COX and its metabolites are involved in various physiological and pathological processes, such as tumour neogenesis, inflammatory response, and blood pressure regulation, and also improve the symptoms of difficult defecation by regulating bowel function. Furthermore, recent studies have reported that COX is involved in developing intestinal motor dysfunction [32]. Inflammation is emerging as a new tip-off to tumours. Elevated levels of COX expression not only inhibit intestinal transport and constipation but can also be a marker of intestinal tumourigenesis. CHRM3 affects the signaling between the synapses of the cholinergic nerves, promotes the contraction of the smooth muscle, and enhances gastrointestinal peristalsis. In addition, core prescriptions can also affect lipids and atherosclerosis, proteoglycans in cancer, hepatitis B, Kaposi's sarcoma-related herpesvirus infection, PI3K-AKTB, and other signaling pathways to regulate the body digestion, circulation, and other systems and the body's metabolism of drugs. It shows that multiple metabolic pathways *in vivo* are involved in the core prescription for constipation treatment mechanism.

The article "Study on Medication Rules of Traditional Chinese Medicine in Treating Constipation through Data Mining and Network Pharmacology" was published in 2022. Journal: Biomed Res Int.

Molecular docking results show that the active ingredients such as quercetin, kaempferol, and stalk flower element bind well with the three target proteins (the binding energy is less than 6 kcal/mol) and have a high matching degree, which reflects good molecular docking, suggesting that the core prescription may play a role through these key targets. These findings may provide further insight into the therapeutic mechanisms of core prescriptions for constipation and may facilitate future screening of potential therapeutic targets.

## 5. Conclusion

This study of prescription medication analysis of constipation through data mining method provides more basis for the treatment of constipation, reduces the difficulty of clinical workers in drug dispensing of constipation treatment, has positive significance for the improvement of clinical efficacy, and makes the continuous improvement of the treatment of constipation in traditional Chinese medicine.

## Figures and Tables

**Figure 1:** Flow chart of research idea.

**Figure 2:** Frequency and efficacy analysis diagram of traditional Chinese medicine. (a) Traditional Chinese medicine with the use frequency of >30 times. (b) The proportion of TCM efficacy classification.

**Figure 3:** Plot of the correlation coefficient of TCM Pearson.

**Figure 4:** Rule chart of TCM association with high-frequency medicine for treating constipation.

**Figure 5:** (a) *K*-means algorithm. (b) PAM algorithm (optimal number of clusters). (c) PAM algorithm (hierarchical clustering dendrograms clustered into 2 classes). (d) GMM algorithm (optimal number of clusters). (e) GMM algorithm (hierarchical clustering dendrograms clustered into 3 classes). (f) GMM algorithm (hierarchical clustering dendrograms clustered into 4 classes).

**Figure 6:** (a) Effective compounds and constipation targets by Venny 2.1. (b) Network of interactions among potential targets of core prescription in the treatment of constipation. (c) Enrichment analysis. (d) Network of “structure types-active ingredients-targets-signal pathways” of the core prescription in treating constipation.

The article "Study on Medication Rules of Traditional Chinese Medicine in Treating Constipation through Data Mining and Network Pharmacology" was published in 2022. Journal: Biomed Res Int.

**Figure 7:** Molecular docking diagram. (a) PTGS1—formononetin. (b) PTGS2—kaempferol. (c) CHRM3—kaempferol.

**Table 1:** TCM order 2 association rules with use frequency >5 times.

No.	Drug pairs			Support	Confidence	Improvement
1	{Dried Rehmanniae Radix}	=>	{Angelicae sinensis Radix}	0.287037	0.805195	1.288312
2	{Semen Persicae}	=>	{Angelicae sinensis Radix}	0.273148	0.808219	1.293151
3	{Ophiopogon japonicas}	=>	{Angelicae sinensis Radix}	0.259259	0.8	1.28
4	{Radix Polygoni multiflori}	=>	{Angelicae sinensis Radix}	0.217593	0.854545	1.367273
5	{Radix Codonopsis}	=>	{Rhizoma Atractylodis macrocephalae}	0.199074	0.895833	1.548
6	{Pericarpium Citri reticulatae}	=>	{Angelicae sinensis Radix}	0.180556	0.829787	1.32766
7	{Radix Achyranthis bidentatae}	=>	{Angelicae sinensis Radix}	0.143519	0.939394	1.50303
8	{Rhizoma cimicifuage}	=>	{Angelicae sinensis Radix}	0.134259	0.805556	1.288889
9	{Radix Rehmanniae preparata}	=>	{Angelicae sinensis Radix}	0.125	0.84375	1.35
10	{Radix Achyranthis bidentatae}	=>	{Cistanche deserticola}	0.125	0.818182	1.767273

**Table 2:** TCM order 3 association rules with use frequency >5 times.

No.	Drug pairs			Support	Confidence	Improvement
1	{Rhizoma Atractylodis macrocephalae, Fructus aurantii}	=>	{Angelicae sinensis Radix}	0.208333	0.8035714	1.28571429
2	{Cistanche deserticola, bitter apricot seed}	=>	{Angelicae sinensis Radix}	0.199074	0.8431373	1.34901961
3	{Rhizoma Atractylodis macrocephalae, bitter apricot seed}	=>	{Angelicae sinensis Radix}	0.199074	0.86	1.376
4	{Rhizoma Atractylodis macrocephalae, Dried Rehmanniae Radix}	=>	{Angelicae sinensis Radix}	0.189815	0.8367347	1.33877551
5	{Radix Glycyrrhizae, Astragali Radix}	=>	{Angelicae sinensis Radix}	0.189815	0.8723404	1.39574468
6	{Cistanche deserticola, Fructus aurantii}	=>	{Angelicae sinensis Radix}	0.185185	0.8695652	1.39130435
7	{Ophiopogon japonicas, Radix Scrophulariae}	=>	{Dried Rehmanniae Radix}	0.180556	0.8125	2.27922078
8	{Dried Rehmanniae Radix, Radix Scrophulariae}	=>	{Ophiopogon japonicas}	0.180556	0.8125	2.50714286
9	{Rhizoma Atractylodis macrocephalae, Ophiopogon japonicas}	=>	{Angelicae sinensis Radix}	0.175926	0.8837209	1.41395349
10	{Cannabis fructus, Cistanche deserticola}	=>	{Angelicae sinensis Radix}	0.175926	0.8636364	1.38181818

**Table 3:** TCM order 4 association rules with use frequency >5 times.

No.	Drug pairs			Support	Confidence	Improvement
1	{Rhizoma Atractylodis macrocephalae, Radix Glycyrrhizae, Astragali Radix}	=>	{Angelicae sinensis Radix}	0.1527778	0.86842105	1.3894737
2	{Angelicae sinensis Radix, Radix Glycyrrhizae, Astragali Radix}	=>	{Rhizoma Atractylodis macrocephalae}	0.1527778	0.80487805	1.3908293
3	{Rhizoma Atractylodis macrocephalae, Cistanche deserticola, bitter apricot seed}	=>	{Angelicae sinensis Radix}	0.1481481	0.84210526	1.3473684
4	{Rhizoma Atractylodis macrocephalae, Astragali Radix, Fructus aurantii}	=>	{Angelicae sinensis Radix}	0.1388889	0.85714286	1.3714286
5	{Angelicae sinensis Radix, Astragali Radix, Fructus aurantii}	=>	{Rhizoma Atractylodis macrocephalae}	0.1388889	0.81081081	1.4010811
6	{Rhizoma Atractylodis macrocephalae, Ophiopogon japonicas, dried Rehmanniae Radix}	=>	{Angelicae sinensis Radix}	0.1342593	0.85294118	1.3647059
7	{Rhizoma Atractylodis macrocephalae, Astragali Radix, dried Rehmanniae Radix}	=>	{Angelicae sinensis Radix}	0.1342593	0.85294118	1.3647059
8	{Angelicae sinensis Radix, Astragali Radix, dried Rehmanniae Radix}	=>	{Rhizoma Atractylodis macrocephalae}	0.1342593	0.82857143	1.4317714
9	{Rhizoma Atractylodis macrocephalae, Cistanche deserticola, Fructus aurantii}	=>	{Angelicae sinensis Radix}	0.1342593	0.85294118	1.3647059
10	{Rhizoma Atractylodis macrocephalae, Radix Glycyrrhizae, Cannabis fructus}	=>	{Angelicae sinensis Radix}	0.1342593	0.82857143	1.3257143

The article "Study on Medication Rules of Traditional Chinese Medicine in Treating Constipation through Data Mining and Network Pharmacology" was published in 2022. Journal: Biomed Res Int.

**Table 4:** The binding energy of component-target.

Component	PTGS1	PTGS2	CHRM3
Kaempferol	-7.22	-8.27	-8.07
Quercetin	-7.63	-7.26	-7.68
Formononetin	-7.72	-7.47	-7.74
Diincarvilone A	-5.98	-6.21	-6.18
Beta-sitosterol	-5.01	-5.25	-5.09

Note: binding energy function [21, 22].

## Data Availability

The datasets used and/or analyzed during the current study are available from the corresponding author on reasonable request.

## Abbreviations

TCM: Traditional Chinese medicine
BC: Betweenness centrality
CC: Closeness centrality
COX-1: Cyclooxygenase-1
COX-2: Cyclooxygenase-2
DC: Degree centrality
DL: Drug-likeness
GO: Gene Ontology
KEGG: Kyoto Encyclopedia of Genes and Genomes
OB: Oral bioavailability
PPI: Protein-protein network
TCMSP: Traditional Chinese Medicine Systems Pharmacology
TCMID: Traditional Chinese Medicine Integrative Database
STRING: Protein-protein interaction networks functional enrichment analysis
DisGeNET: A database of gene-disease association
GeneCards: Human genes, protein and diseases
PTGS2: Prostaglandin-endoperoxide synthase 2
PTGS1: Prostaglandin-endoperoxide synthase 1
CHRM3: Recombinant cholinergic receptor, muscarinic 3
PI3K/AKT: Phosphatidylinositol 3-kinase and protein kinase B.
